This article has been retracted.

# Analysis of Serum Levels of IFN-*γ*, IL-4, and TNF-*α* in Patients with Cervicitis Complicated by HPV Infection and Their Clinical Significance

**DOI:** 10.1155/2022/3374655

**Published:** 2022-04-13

**Authors:** Jingxia Li, Yuejun Liu, Jianjun Song, Wenli Liu, Liyuan Zhou, Shucheng Chen

**Affiliations:** ^1^Gynecology Department, Affiliated Hospital of Hebei University of Engineering, Handan 056000, Hebei, China; ^2^Gynecology Department, Fourth Affiliated Hospital of Hebei Medical University, Shijiazhuang 050000, Hebei, China

## Abstract

In order to investigate the expression levels of serum IFN-*γ*, IL-4, and tumor necrosis TNF-*α* in patients with cervicitis complicated with human papillomavirus (HPV) infection and clinical significance, a retrospective study was conducted on 90 patients with chronic cervicitis complicated by HP V infection who visited our hospital from June 2020 to June 2021, and they are included in the research group. According to the degree of HPV infection, the patients are divided into low-risk HPV type group (*n* = 65 cases) and high-risk HPV type group (*n* = 25 cases); 50 patients with cervicitis (without HPV infection) who received treatment in our hospital are selected as control group 1. Fifty healthy women who underwent physical examination are selected as the control group 2. The general data of the two groups of patients during hospitalization are collected, and HPV-DNA, IFN-*γ*, IL-4, and TNF-*α* are detected in all patients. For patients with cervicitis complicated by HPV infection, the IFN-indexes in the body are significantly decreased, IL-4 and TNF-*α*are significantly increased, and with the degree of HPV infection, IFN-*γ*, IL-4, and TNF-*α* have high diagnostic performance with HPV infection, and there is a significant correlation between the three, which can be used in cervicitis complicated with HPV infection. It is widely used in the early diagnosis and screening of infected patients.

## 1. Introduction

Cervical disease is a common disease in women of childbearing age, generally including acute and chronic cervicitis, cervical intraepithelial neoplasia CIN, and cervical cancer [1]. Among them, cervicitis is a common gynecological disease in clinical cervical diseases. Because most of the patients are women of childbearing age, its pathogenesis is mainly related to childbirth, miscarriage, and frequent sexual life [2]. Relevant studies have found that there is a significant correlation between human papillomavirus (human papilloma virus, HPV) infection and the occurrence of cervicitis. Usually, HPV infection in patients with cervicitis has a higher carcinogenic rate. It can lead to the occurrence of cervical cancer and pose a serious threat to the health of patients [3]. Therefore, early diagnosis of chronic cervicitis is extremely important. Once cervicitis occurs in clinical patients, the main clinical manifestations are genital itching, lumbosacral pain, increased vaginal secretions, or purulent secretions, etc. If the patient is not treated in time, the disease will be allowed to develop and will further develop into cervical hypertrophy, cervical erosion, and other serious cervical diseases. Studies have shown that HPV infection is a high-risk factor for cervicitis, and chronic cervicitis combined with HPV infection, especially persistent high-risk HPV infection, is a high-risk factor for cervical cancer [4]. Under normal circumstances, the ectopic surface of the cervical columnar epithelium is composed of a single layer of a tall columnar epithelium and secretes a protective mucus, but the ectopic cervical columnar epithelium is easily stimulated by vaginal inflammatory factors, resulting in thinning of the genital tract mucosa and reduced protective mucus secretion. It is the best channel to increase the chance of HPV infection [5]. About 90% of cervical cancer specimens can detect HPV virus genes or gene fragments, and whether the persistent infection of HPV in the human body can cause cervical lesions is closely related to the infected person's own state and immune system regulation. There is a close relationship between immune regulation and HPV-mediated carcinogenesis, and there is a significant correlation between the two [6].

In order to investigate the expression levels of serum IFN-*γ*, IL-4, and tumor necrosis TNF-*α* in patients with cervicitis complicated with human papillomavirus (HPV) infection and clinical significance, this paper selects patients with cervicitis complicated by HPV infection to analyze the interferon*γ* (interferon gamma) in vivo. The expression levels of IFN-*γ*, IL-4, and TNF-*α* are analyzed and their correlation with HPV infection is analyzed.

## 2. Methodology

### 2.1. General Information

90 patients with chronic cervicitis complicated by HPV infection who were treated in our hospital from June 2020 to June 2021 were retrospectively selected and included in the research group. According to the degree of HPV infection, the patients are divided into low-risk HPV type group (*n* = 65 cases) and high-risk HPV type group (*n* = 25 cases); 50 patients with cervicitis (without HPV infection) who received treatment in hospital are selected as control group 1. 50 healthy women served as the control group 2. Among them, the age of the patients in the study group is in the range of 23–58 years old, with an average of (42.49 ± 9.82) years old; in 1 to 4 times of pregnancy, with an average of (1.81 ± 1.03) times, the disease duration is 3 months to 55 months, with an average of (22.93 ± 11.76) months. Control group 1: aged from 23 to 59 years old, with an average of (42.86 ± 9.69) years old; in 0 to 5 times of pregnancy, with an average of (1.80 ± 0.97) times, the disease duration is 5 months to 55 months, with an average of (23.32 ± 12.74) months. Control group 2: aged 23 to 58 years, mean (41.64 ± 7.88) years old; 0 to 5 pregnancies, mean (1.82 ± 1.10) times. Comparing the general basic data such as age and course of disease among the three groups, there is no significant difference which can be compared (*P* > 0.05).

### 2.2. Inclusion and Exclusion Criteria

Inclusion criteria were as follows: (1) met the diagnostic criteria for cervicitis in Obstetrics and Gynecology (8th Edition) [7]; (2) the result of liquid-based cytology test is positive [8]; (3) there is a history of sexual life [9–11]; and (4) age ≥ 18 years old.

The exclusion criteria include the following eight aspects: (1) cervical epithelial neoplasia grade II to III; (2) diagnosed with early cervical cancer or combined with other types of malignant tumors; (3) presence of trichomoniasis, candida, and other reproductive system infections; (4) combined with heart and brain patients with a vascular disease or dysfunction; (5) diagnosed with autoimmune or blood diseases; (6) taking hormone- related drugs or immunotherapy within the past 3 months; (7) history of pelvic radiation therapy; and (8) be pregnant or breastfeeding.

The general data of the two groups of patients during hospitalization are collected, including age, course of disease, pregnancy, and other related indicators [12–15]. In the bladder lithotomy position of the patient, the cervical secretions are wiped off with a dry cotton ball, and the cervical brush is inserted into the internal cervical orifice through the HPV sampler, attached to the mucosa of the transition zone, and rotated counterclockwise for 4 weeks. DNA is extracted from the lysate, and HR-HPV genotypes are detected by the second-generation hybrid capture technology (HC2), including HPV 16, 18, 31, 33, 35, 39, 45, 51, 52, 56, 58, 59, 66, and 68 The results are expressed as the ratio of relative luminescence value (RLU) measured by a specimen fluorometer to a positive calibration threshold value (CO), RLU/CO ≥ 1.0 represents a positive result, which is equivalent to the DNA load detected in the specimen ≥ 1.0 pg/ml, RLU/CO < 1.0 means negative.

5 ml of cubital venous blood is drawn from all the participating research subjects on an empty stomach in the morning, 3 500 r/min, about 10 min, and the centrifugation radius is 10 cm. The serum IFN-*γ* and IL-4 levels are detected using an ELISA kit; it is purchased from TSZ in the United States. The standard curve is drawn and the corresponding concentrations are calculated [10, 11, 16–19]. The TNF-alpha level is also calculated. The abovementioned operations are all carried out by the same researcher, and the operations are carried with the kit.

All data are summarized and sorted, and a database is established for all data. Using SPSS 24.0 software, normality and homogeneity of variance are tested to satisfy normal distribution. The differences tested are considered statistically significant.

## 3. Experimental Results

### 3.1. Expression Levels of Serum in the Study Group and the Control Group

In terms of IFN-*γ* levels, the study group is the lowest and the control group 2 is the highest; IL-4 and TNF-*α* levels are the lowest in the study group and the highest in the control group 2(both *P* < 0.05).  Table 1 shows serum expression levels in study group and control group.

### 3.2. Expression Levels of Serum in High-Risk and Low-Risk HPV Groups

From the level of IFN-*γ* index, the group with high HPV infection is significantly higher, and from the level of IL-4 and TNF-*α*, the group with high HPV infection is significantly lower, both of which are related to the group with low HPV infection. Compared with the group, all *P* < 0.05..  Table 2 shows expression levels of serum in the high-risk HPV group and low-risk HPV group.

### 3.3. Correlation between Cervicitis Complicated with HPV Type Infection and the Expression

Cervicitis combined with HPV type infection is significantly negatively correlated with IFN-*γ* (*r* = −0.846, *P* < 0.001); cervicitis combined with HPV type infection is significantly positively correlated with both IL-4 and TNF-*α* ((*r* = 0.798, 0.853), all *P* < 0.001).  Table 3 shows the correlation between cervicitis complicated with HPV type infection and the expression of IFN-*γ*, IL-4, and TNF-*α*.

### 3.4. Diagnostic Value of Cervicitis Complicated with HPV Infection

#### 3.4.1. Diagnostic Value of Patients with High-Risk HPV Infection

The area under the ROC curve of IFN-*γ*, IL-4, and TNF-*α* for the assessment of high-risk HPV infection, all exceeded 0.75, which had high specificity and sensitivity. There is no statistical difference in the prediction models of the three detection methods.  Table 4 displays the diagnostic value of patients with high-risk HPV infection.  Figure 1 shows the ROC curve of the diagnostic value of patients with high-risk HPV infection.

#### 3.4.2. Diagnostic Value of in Patients with Low-Risk HPV Infection

The area under the ROC curve of IFN-*γ*, IL-4, and TNF-*α* for the assessment of low-risk HPV infection, all exceeded 0.75, which had high specificity and sensitivity. There is no statistical difference in the prediction models of the three detection methods.  Table 5 shows the diagnostic value of patients with low-risk HPV infection.  Figure 2 presents the ROC curve of the diagnostic value of patients with low-risk HPV infection.

### 3.5. Correlation Analysis of Expression in Patients with Cervicitis Complicated by HPV

From the correlation of different serum indexes, there is a significant correlation among the three, and IFN-*γ* is significantly negatively correlated with IL-4 and TNF-*α* (*r* = −0.803). There is a significant positive correlation with TNF-*α* (*r* = 0.870) (both *P* < 0.05).  Figure 3 shows the correlation analysis of expression in patients with cervicitis complicated by HPV.

## 4. Assessment and Testing

Chronic cervicitis is one of the most common diseases in clinical gynecology. According to statistics, about 60% of married women suffer from chronic cervicitis of varying degrees. In severe cases, infertility may occur, which is the main reason for patients to seek medical treatment. It not only poses a major threat to female reproductive health but also seriously affects the mental health of patients. It is well known that chronic cervical inflammation is closely related to cervical carcinoma and its mortality rate ranks first in gynecological cancer. 130,000 new cases of cervical cancer increase in my country every year, accounting for more than 1/4 of the world, and the trend of younger patients is obvious, which has caused a huge impact and damage to the body and mind of patients. For most women, it is a relatively long process from chronic cervicitis to cervical precancerous lesions to cervical cancer, and early intervention and treatment are extremely important and achievable for the prevention of cervical cancer. Therefore, the treatment of chronic cervical inflammation and the eventual eradication of cervical cancer will become the main issues for women in our country and the world to overcome serious diseases and benefit women's health. Studies have found that HPV infection has an important relationship with cervicitis. The infection of HPV in patients with cervicitis has a high carcinogenic rate, which can lead to cervical cancer and pose a serious threat to the health of patients. However, whether or not persistent HPV infection can cause the occurrence and development of cervical lesions, it is related to factors such as the autoimmune state and hormone secretion level of the infected person, and the host autoimmune regulation plays a key role in HPV-mediated carcinogenesis.

This study found that the levels of IFN-*γ* in different groups of patients showed different differences (all *P* < 0.05). Tumor and immunomodulatory effects can prevent or slow the transformation of normal cells to tumor cells, and abnormal levels of IFN-*γ* may lead to tumorigenesis. Zhang Jing detected the expression of IFN-*γ* in the tissues of cancer patients and showed that the expression of IFN-*γ* in cancer tissues is lower than that in surrounding normal tissues and in the later tumor stage, the IFN-*γ* level is lower. IL-4 is a major cytokine that can inhibit the response of Th1-type cytokines and mediate the development of Th2-type cells, which is closely related to tumor malignancies. Luo et al. detected the peripheral blood mononuclear cells of breast cancer patients and the culture supernatant to detect the level of IL-4 and found that the level of IL-4 in breast cancer patients is higher than that in the normal control group, which has a markedly different significance (*P* < 0.05). Yu also analyzed the IL-4 concentration in the peripheral blood culture supernatant of cervical cancer patients and found that the IL-4 concentration in the peripheral blood mononuclear cell culture supernatant of cervical cancer patients is comparable to normal examination. The study detected IL-4 in patients with cervicitis complicated by HPV infection and found that with the aggravation of HPV type infection (*P* < 0.01). High IL-4 levels may indicate another malignant trend of the disease, suggesting that patients have more severe cervical lesions, and the more obvious the local immunosuppression, the easier it is for cancer cells to escape immune surveillance and accelerate tumor progression. In addition, statistical analysis found that IFN-*γ* and IL-4 concentrations are negatively correlated, suggesting that IFN-*γ*gradually decreased, IL-4 gradually increased, and IFN-*γ*/IL-4 gradually increased, which can more intuitively explain the two indicators. This study also found that cervicitis combined with HPV type infection is significantly negatively and IFN-*γ* (*r* = -0.846, *P* < 0.001); cervicitis combined with HPV type infection is significantly positively correlated with both IL-4 and TNF-*α* (both *P* < 0.001); TNF-*α*is a pleiotropic cytokine, which is mainly secreted by macrophages and is widely involved in the process of cellular reactions. When the human body has fever, shock, tissue damage, and tumor necrosis When the effect is equating-*α* can be induced by other cytokines and immunoregulatory factors, making it involved in cell proliferation, differentiation, and apoptosis. In addition, TNF-*α* can bind to receptors on the surface of cancer cells, and after the complexation is completed, it enters the cell and fuses with the lysosome. At this time, TNF-*α* plays an important role, which will promote the lysis of lysosomes and the release of proteases, and then cause cell autolysis. Although this study has achieved certain results, due to the relatively small number of cases included in the study, it may cause a certain bias to the results. Therefore, the sample size needs to be further expanded in future studies to further analyze the serum levels of IFN-*γ* and IL-4 in patients with cervicitis complicated by HPV infection.

## 5. Conclusion

This paper selects patients with cervicitis complicated by HPV infection to analyze the interferon*γ* (interferon gamma) in vivo. The expression levels of IFN-*γ*, IL-4, and TNF-*α* are analyzed, and their correlation with HPV infection is analyzed. The IFN-*γ* indexes in patients with cervicitis complicated with HPV infection are significantly decreased and those of IL-4 and TNF-*α* are significantly increased. IL-4 and TNF-*α* have a high diagnostic performance with HPV infection, and there is a significant correlation between the three, which can be widely used in the early diagnosis and screening of patients with cervicitis complicated with HPV infection.

## Figures and Tables

**Figure 1:** ROC curve of diagnostic value of patients with high-risk HPV infection.

**Figure 2:** ROC curve of the diagnostic value of patients with low-risk HPV infection.

**Figure 3:** Correlation analysis of expression in patients with cervicitis complicated by HPV.

**Table 1:** Serum expression levels in study group and control group.

Group	Number of cases (*n*)	IFN-*γ* (pg/ml)	IL-4 (pg/ml)	TNF-*α* (*μ*g/L)
Research group	90	85.61 ± 11.58∗#	96.92 ± 13.80^∗#^	12.70 ± 1.89^∗#^
Control group 1	50	96.35 ± 5.88#	86.69 ± 5.65^#^	8.93 ± 0.84^#^
Control group 2	50	103.26 ± 5.95	75.97 ± 5.21	2.62 ± 0.74
*F*		−11.296	9.872	12.596
*P*		<0.001	<0.001	<0.001

**Table 2:** Expression levels of serum in the high-risk HPV group and low-risk HPV group.

Group	Number of cases (*n*)	IFN-*γ* (pg/ml)	IL-4 (pg/ml)	TNF-*α* (*μ*g/L)
High-risk HPV group	25	82.81 ± 4.92	103.54 ± 9.92	13.69 ± 0.98
Low-risk HPV group	65	92.88 ± 5.33	79.70 ± 3.40	10.14 ± 1.11
*t*		−8.195	17.063	14.018
*P*		<0.001	<0.001	<0.001

**Table 3:** Correlation between cervicitis complicated with HPV type infection and the expression of IFN-*γ*, IL-4, and TNF-*α*.

	HPV type infection	
	*r*	*P*
IFN-*γ*	−0.846	<0.001
IL-4	0.798	<0.001
TNF-*α*	0.853	<0.001

**Table 4:** Diagnostic value of patients with high-risk HPV infection.

Index	Accuracy	Sensitivity	Specificity	AUC
IFN-*γ*	82.00	65.50	75.26	0.775 (0.564∼0.893)
IL-4	72.00	80.00	78.60	0.795 (0.662∼0.857)
TNF-*α*	76.00	78.50	75.20	0.782 (0.613∼0.873)

**Table 5:** Diagnostic value of patients with low-risk HPV infection.

Index	Accuracy	Sensitivity	Specificity	AUC
IFN-*γ*	76.00	80.50	70.26	0.761 (0.692∼0.863)
IL-4	78.00	80.00	78.60	0.794 (0.696∼0.847)
TNF-*α*	75.00	77.50	75.00	0.779 (0.713∼0.869)

## Data Availability

The simulation experiment data used to support the findings of this study are available from the corresponding author upon request.
